The article "Plexin-B1 Activates NF-κB and IL-8 to Promote a Pro-Angiogenic Response in Endothelial Cells" was retracted in 2019. Reason: duplicated images.

# Plexin-B1 Activates NF-κB and IL-8 to Promote a Pro-Angiogenic Response in Endothelial Cells

**DOI:** 10.1371/journal.pone.0025826

**Published:** 2011-10-18

**Authors:** Ying-Hua Yang, Hua Zhou, Nada O. Binmadi, Patrizia Proia, John R. Basile

**Affiliations:** 1 Department of Oncology and Diagnostic Sciences, University of Maryland Dental School, Baltimore, Maryland, United States of America; 2 Department of Sports Science (DISMOT), University of Palermo, Palermo, Italy; 3 Marlene and Stuart Greenebaum Cancer Center, Baltimore, Maryland, United States of America; Fundação Oswaldo Cruz, Brazil

## Abstract

**Background:**

The semaphorins and their receptors, the plexins, are proteins related to c-Met and the scatter factors that have been implicated in an expanding signal transduction network involving co-receptors, RhoA and Ras activation and deactivation, and phosphorylation events. Our previous work has demonstrated that Semaphorin 4D (Sema4D) acts through its receptor, Plexin-B1, on endothelial cells to promote angiogenesis in a RhoA and Akt-dependent manner. Since NF-κB has been linked to promotion of angiogenesis and can be activated by Akt in some contexts, we wanted to examine NF-κB in Sema4D treated cells to determine if there was biological significance for the pro-angiogenic phenotype observed in endothelium.

**Methods/Principal Findings:**

Using RNA interference techniques, gel shifts and NF-κB reporter assays, we demonstrated NF-κB translocation to the nucleus in Sema4D treated endothelial cells occurring downstream of Plexin-B1. This response was necessary for endothelial cell migration and capillary tube formation and protected endothelial cells against apoptosis as well, but had no effect on cell proliferation. We dissected Plexin-B1 signaling with chimeric receptor constructs and discovered that the ability to activate NF-κB was dependent upon Plexin-B1 acting through Rho and Akt, but did not involve its role as a Ras inhibitor. Indeed, inhibition of Rho by C3 toxin and Akt by LY294002 blocked Sema4D-mediated endothelial cell migration and tubulogenesis. We also observed that Sema4D treatment of endothelial cells induced production of the NF-κB downstream target IL-8, a response necessary for angiogenesis. Finally, we could show through co-immunofluorescence for p65 and CD31 that Sema4D produced by tumor xenografts in nude mice activated NF-κB in vessels of the tumor stroma.

**Conclusion/Significance:**

These findings provide evidence that Sema4D/Plexin-B1-mediated NF-κB activation and IL-8 production is critical in the generation a pro-angiogenic phenotype in endothelial cells and suggests a new therapeutic target for the anti-angiogenic treatment of some cancers.

## Introduction

The semaphorins are a family of secreted, transmembrane and glycosylphosphatidylinositol-linked proteins characterized by large cysteine-rich semaphorin domains that were originally identified based on their ability to provide both attractive and repulsive axon guidance cues during neural development [1]. They are now known to be expressed in tissues outside of the nervous system where they are involved in many motility responses including regulation of cell-cell contacts and branching morphogenesis in epithelium [2], promotion of angiogenesis [3], [4], and growth and metastasis of tumors [5], [6]. The main functional receptors for semaphorins are a family of single pass transmembrane proteins known as plexins [7], [8]. The intracellular portion of the plexins contain a GTPase-activating protein (GAP)-like motif that downregulates activity of the G protein R-Ras, interrupted by a region capable of binding small Rho family GTPases [9], [10]. In the case of Plexin-B1 for example, this Rho GTPase binding domain (RBD) can associate with Rnd1, Rac1, and RhoD, the binding of which influences plexin functioning [10]. The small GTPases act as molecular switches that cycle between an active GTP-bound and inactive GDP-bound form to regulate microtubule dynamics, cell shape and cell mobility [11]. Therefore, it is likely that the binding of semaphorins to plexins initiates a signaling cascade that impinges upon the cytoskeleton [12]. In addition to the small GTPases, kinase activity plays a vital role in plexin signaling. The plexins themselves are devoid of any intrinsic kinase activity, so this function is provided by kinases activated by the signaling complex, depending upon the class of plexins and the context.

The nuclear factor (NF)-κB family of transcription factors plays an important role in the ability of a cell to adapt to environmental changes and figures prominently in many biological processes. NF-κB dimers positively or negatively regulate expression of target genes in response to bacterial products, cytokines, viral infection, growth factors and other stressful stimuli [13]. In the inactive form, NF-κB is bound to the inhibitor of κB (I-κB) family of proteins that sequester NF-κB dimers in the cytoplasm. Upon stimulation, the I-κB kinase (IKK) complex phosphorylates the I-κB proteins on two conserved N-terminal serine residues, which target them for E2- and E3-ligase-mediated polyubiquitination and subsequent 26S proteasomal degradation [14]. This process releases and activates NF-κB, freeing it up to move to the nucleus where it undergoes a series of posttranslational modifications and binds to specific DNA sequences in target genes (designated as “κB elements”) that regulate the transcription of over 500 genes involved in inflammation, the immune response, cell growth control and the regulation of cell survival [14]. Importantly, dysregulated NF-κB activity has been associated with tumor promotion, suppression of apoptosis, tumor-induced angiogenesis and metastasis [15].

Our lab and others have shown that Semaphorin 4D (Sema4D) is pro-angiogenic when acting through its receptor Plexin-B1 on endothelial cells [3], [4] and may be produced by malignancies for the purposes of promoting blood vessel growth into the tumor [16]. There is a PDZ binding motif at the C-terminus of Plexin-B1 that associates with PDZ-Rho guanine nucleotide exchange factor (GEF) and leukemia-associated RhoGEF (LARG), proteins that activate Rho [17], [18]. Sema4D binding to Plexin-B1 also promotes Rnd1-dependent activation of receptor GAP activity and R-Ras inhibition [9], [10]. Finally, there is evidence that Plexin-B1 competes with p21-activated kinase (PAK) for Rac binding, sequestering the active form of Rac and inhibiting Rac-dependent processes [19]. We previously have demonstrated that pro-angiogenic Plexin-B1 signaling is dependent upon its ability to activate Rho, specifically by signaling through the downstream effector Rho kinase (ROK) and activating Akt, Src and Pyk2 [20].

Since NF-κB has been linked to promotion of angiogenesis in some malignancies [21] and IKK can be phosphorylated by Akt, leading to activation of NF-κB [22], we wanted to examine NF-κB in response to Plexin-B1 stimulation and determine if there was any biological significance for the pro-angiogenic phenotype observed in endothelial cells. Here we show that NF-κB and its pro-angiogenic effector IL-8 are activated downstream of Plexin-B1. In endothelial cells, this response occurred following treatment with Sema4D and was necessary for chemotaxis, capillary tube formation and resistance to apoptosis. We could elicit NF-κB activation in endothelial cells when treated by conditioned media from head and neck squamous cell carcinoma (HNSCC) cell lines expressing Sema4D and demonstrate activation of NF-κB *in vivo* in a tumor xenograft model. Taken together, these results demonstrate further versatility in plexin signaling that may hint at new diagnostic and therapeutic approaches in the anti-angiogenic treatment of some cancers.

## Results

### Sema4D activates NF-κB through Plexin-B1

Though Sema4D is also known to bind to lower-affinity receptors such as CD72 (on cells of hematopoietic origin, which include endothelial cells) [23] and Plexin-B2 (which has only been observed in neurons) [24], we previously have demonstrated that promotion of a pro-angiogenic phenotype in endothelial cells is due to ligation by Sema4D of its high-affinity receptor, Plexin-B1 [4], which in turn activates Akt [25]. The pro-inflammatory and pro-cell survival protein NF-κB is a known functional target of Akt [22], [26] and has been linked to angiogenesis. Therefore, we wanted to look for Plexin-B1-mediated NF-κB activation in Sema4D treated endothelial cells. NF-κB is sequestered in the cytoplasm by I-κB, which needs to be phosphorylated and degraded to allow NF-κB to translocate to the nucleus, so rapid phosphorylation and loss of I-κB signal in an immunoblot (and then recovery, as I-κB is induced by NF-κB) is a good marker for activation of NF-κB. To determine the role of Plexin-B1 in the activation of NF-κB, we infected HUVEC with control lentivirus or lentivirus coding for Plexin-B1 shRNA and confirmed protein knockdown in an immunoblot (Figure 1A). We then treated these cells with 400 ng/ml Sema4D and observed I-κB phosphorylation (Figure 1B, upper panel, left) and degradation (Figure 1B, middle panel, left), but loss of this response in cells expressing reduced levels of Plexin-B1 (Figure 1B, right panels). We treated control cells and those infected with Plexin-B1 shRNA-expressing lentivirus with soluble Sema4D, lysed them and incubated the nuclear fraction with labeled oligonucleotides containing κB elements to look for binding in an electrophoretic mobility shift assay. NF-κB binding was detected by a gel shift in Sema4D treated cells but not in cells infected with Plexin-B1 shRNA (Figure 1C). Specificity of this assay was demonstrated by a supershift upon incubation with a p65 antibody and a loss of signal when incubated with a 100-fold excess of unlabelled oligonucleotide (Figure 1C). We also detected the NF-κB subunit p65 migrating to the nucleus in an immunofluorescence analysis of Sema4D treated HUVEC (Figure 1D) and in an immunoblot of nuclear and cytoplasmic fractions from these cells (Figure 1E). We then looked for NF-κB activation in a reporter assay in HUVEC expressing an NF-κB responsive luciferase construct, following treatment with Sema4D. We observed a concomitant increase in fluorescence with increasing concentrations of Sema4D (Figure 1F). Taken together, these results demonstrate that Sema4D induces NF-κB translocation to the nucleus and transcriptional activity in endothelial cells in a Plexin-B1-dependent manner.

**Figure 1:** Sema4D activates NF-κB downstream of Plexin-B1. A. Immunoblot analysis for Plexin-B1 on lysates from endothelial cells infected with empty vector control lentivirus (control) or virus coding for Plexin-B1 shRNA (PB1shRNA). GAPDH was used as a loading control (lower panel). B. Immunoblot for phospho- and total I-κB (upper and middle panels, respectively) in endothelial cells infected with empty vector control lentivirus (control, left column) or virus coding for Plexin-B1 shRNA (PB1shRNA, right column) treated with Sema4D for the times indicated. GAPDH was used as a loading control (lower panels). C. EMSA performed on control infected HUVEC or cells infected with lentivirus coding for Plexin-B1 shRNA, in the presence of Sema4D with and without competition from unlabeled oligos (competition) or anti-p65 antibody (p65 antibody). “ns” denotes a non-specific band; “NF-κB” indicates a shift in oligo migration; “supershift” indicates the higher band resulting from antibody binding. D. Immunofluorescence for the presence of the p65 subunit of NF-κB in nuclei of HUVEC, controls (top row) or treated with Sema4D (bottom row). p65 is shown in green (center column). DAPI was used to stain cell nuclei (left column). The merged image is shown in the right column. E. Immunoblot for the presence of p65 in cytoplasmic and nuclear fractions of HUVEC treated with Sema4D. GAPDH was used as a loading control (lower panel). F. HUVEC were infected with lentiviruses coding for an NF-κB reporter construct and fluorescence measured in arbitrary units (AU) in increasing concentrations of Sema4D, as indicated. Error bars represent the standard deviation from three experiments.

### Sema4D induces a pro-angiogenic phenotype and apoptotic protection in endothelial cells through NF-κB but has no effect on proliferation or VEGF-mediated angiogenesis

To determine the biological significance of the activation of NF-κB we observed in endothelial cells, we performed a Boyden chamber migration assay on HUVEC, as an *in vitro* measure of angiogenesis, with and without the NF-κB inhibitor BAY11-7085 and an I-κB mutant protein resistant to phosphorylation and degradation (the “super-repressor”), using Sema4D as the chemoattractant. HUVEC migrated towards Sema4D, as we and others have observed before [3], [4], except when co-treated with BAY11-7085 (Figure 2A), and where cells were infected with lentiviruses coding for the I-κB super-repressor (Figure 2B, results quantified for both migration assays in the bar graph, lower panels). HUVEC continued to migrate towards FBS in both instances, indicating the specificity of NF-κB activation in Sema4D-mediated chemotaxis. We also looked for the ability of these cells growing on reconstituted basement membrane material to form tube-like capillary structures in tissue culture under similar conditions, which is indicative of a pro-angiogenic response. HUVEC formed capillary tubes when growing on reconstituted basement membrane material in the presence of Sema4D except when co-treated with BAY11-7085 (Figure 2C) or when expressing the I-κB super-repressor (Figure 2D, results quantified for both tubulogenesis assays in the bar graph, lower panels). NF-κB is also known to promote cell survival and proliferation in different cell lines. In order to determine the effects of Sema4D-mediated activation of NF-κB on endothelial cell survival, we treated HUVEC with soluble Sema4D and looked for resistance to apoptosis under conditions of serum starvation, with or without the NF-κB inhibitor BAY 11-7085. We noted the presence of cleaved, and hence activated, caspase 3 in serum starved cells, a response which decreased in increasing concentrations of Sema4D but returned when the cells were co-treated with BAY 11-7085, indicating that this effect was dependent upon Sema4D-induced NF-κB activity (Figure 2E). To evaluate if endothelial cell proliferation is enhanced by Sema4D, we measured HUVEC proliferation by [^3^H] thymidine incorporation assay, using vascular endothelial growth factor (VEGF) treatment as a positive control. As expected, VEGF treated HUVEC were stimulated to proliferate, incorporating [^3^H] at three times the rate of controls (Figure 2F). Interestingly, no concentrations of Sema4D seemed to influence HUVEC proliferation (Figure 2F).

**Figure 2:** Sema4D induces migration, capillary tube formation and apoptotic protection in endothelial cells in an NF-κB-dependent manner, but has no effect on endothelial cell proliferation or VEGF-mediated angiogenesis. A. Migration assays on HUVEC towards BSA, FBS or Sema4D in the presence of control media or media containing BAY11-7085 (BAY). B. Migration assays on HUVEC, control infected (C), or infected with the I-κB super-repressor (SR) towards BSA, FBS or Sema4D. C. HUVEC treated with vehicle control (neg ctrl), or BAY11-7085 (BAY), with or without Sema4D were grown on reconstituted basement membrane material in serum free media and examined for formation of capillary tubes. Representative photographs are shown. D. HUVEC mock electroporated (mock), or electroporated with the I-κB super-repressor (SR) were grown on reconstituted basement membrane material in serum free media with or without Sema4D and examined for formation of capillary tubes. Representative photographs are shown. E. Immunoblot performed for the cleaved fragment of caspase 3 (top panel) in HUVEC growing under conditions of low serum concentration, treated with the indicated concentrations of Sema4D with or without the NF-κB inhibitory compound BAY11-7085 (BAY). GAPDH was used as a loading control (lower panel). F. An [^3^H] thymidine incorporation assay was performed on HUVEC growing in the presence of Sema4D or VEGF for the purposes of measuring proliferation. Counts per minute (cpm) are represented on the Y-axis. Error bars represent the standard deviation from four independent experiments. G. Migration assay on HUVEC, control infected (control), or infected with lentiviruses expressing Plexin-B1 shRNA (Plexin-B1 shRNA) towards BSA, Sema4D or VEGF. For all migration assays, the results are quantified by the bar graphs in the bottom panels as the pixel intensity of scanned migration assay membranes, which are shown on the top. Error bars represent the standard deviation from six wells (*, p<0.05; n.s., not significant). H. HUVEC, control infected (control), or infected with lentiviruses expressing Plexin-B1 shRNA (Plexin-B1 shRNA) were grown on reconstituted basement membrane material in serum free media with BSA, Sema4D or VEGF and examined for formation of capillary tubes. Representative photographs are shown. Quantification of the results of all tubulogenesis assays are shown in the bar graphs in the lower panels, with the Y-axis representing tube formation as measured by summing the length of capillary tubular structures observed in 10 microscopic fields, relative to the negative control wells (error bars represent the standard deviation from three independent experiments; *, p<0.05; n.s., not significant).

Because we noted endothelial cell proliferation in the presence of VEGF but not Sema4D, we suspected that these two pro-angiogenic factors elicited different signaling pathways and possibly functioned independently of each other. To further establish their independence and evaluate the role of Sema4D and Plexin-B1 in the broader context of the angiogenic process, we performed *in vitro* angiogenesis assays on endothelial cells, with and without silenced Plexin-B1, in the presence of Sema4D and VEGF, and compared the responses. Sema4D and VEGF induced robust endothelial cell migration compared to control populations (Fig. 2G). Sema4D-mediated cell migration was greatly reduced in cells infected with lentiviruses expressing Plexin-B1 shRNA, while migration toward VEGF remained unaffected (Figure 2G, results quantified in the bar graph, lower panel). We then confirmed these results in a tubulogenesis assay, growing endothelial cells on reconstituted basement membrane extract under the same conditions. Once again, HUVEC formed capillary tube-like structures when growing in the presence of Sema4D except when infected with Plexin-B1 shRNA-expressing lentivirus, while cells growing in VEGF formed these structures regardless of their Plexin-B1 status (Figure 2H, results quantified in the bar graph, lower panel).

Taken together, these findings indicate that NF-κB activation is necessary for the Sema4D-mediated pro-angiogenic phenotype in endothelial cells. This response is probably due to endothelial cell chemotaxis and differentiation into capillary structures and not due to an effect on cell proliferation, unlike what was observed for VEGF. Furthermore, insensitivity of endothelial cells to Plexin-B1 status in the presence of VEGF suggests that Sema4D and VEGF work through independent, parallel pathways to achieve their respective pro-angiogenic responses.

### RhoA and Akt are necessary for Plexin-B1-mediated activation of NF-κB and promotion of endothelial cell migration and tube formation by Sema4D

To dissect the pathways involved in Plexin-B1-mediated NF-κB activation, and to rule out involvement of CD72 or Plexin-B2 in this process, we looked for phosphorylation and degradation of I-κB in cells expressing plasmids coding for the chimeric receptors TrkA fused to full length Plexin-B1, Plexin-B1 lacking the C-terminal PDZ binding domain necessary to activate Rho, and a chimera containing Plexin-B1 with mutations at the arginine residues required for R-RasGAP activity [4], [17]. We have previously shown that we could isolate and study Plexin-B1 specific signaling in cells expressing these constructs when treated with NGF [4], [17]. We also co-treated with the Rho inhibitor C3 toxin or the PI3K inhibitor LY294002, where indicated, in order to clarify further the role of Ras, Rho and Akt in the NF-κB response. Phosphorylated I-κB was observed in control treated cells transfected with the full-length chimera, which was then rapidly degraded as expected (Figure 3A). However, this response was absent in cells expressing the full-length chimera but incubated with C3 or LY294002 and in all cells expressing the ΔPDZ chimera incapable of activating Rho (Figure 3A). The R-RasGAP mutant was still able to elicit phosphorylation and degradation of I-κB except when co-treated with C3 or LY294002, indicating that this effect was independent of R-RasGAP activity (Figure 3A). To further confirm the role of Rho and Akt in this process, we looked for activation of NF-κB transcription in a reporter assay in HUVEC transfected with an NF-κB responsive luciferase construct, treated with Sema4D with and without C3 or LY294002. Fluorescence was greatly increased in Sema4D treated HUVEC except when co-treated with C3 or LY294002 (Figure 3B). We then evaluated the ability of HUVEC to exhibit chemotaxis or form capillary tube structures in Sema4D, with or without Rho and Akt inhibition. HUVEC migrated towards Sema4D, a response that was blocked by C3 and LY294002 (Figure 3C, results quantified in the bar graph, lower panel), and could form tubes on reconstituted basement membrane material in the presence of Sema4D except when co-incubated with C3 or LY294002 (Figure 3D, results quantified in the bar graph, right panel). Taken together, these results indicate that Plexin-B1 activates NF-κB in a Rho and Akt-dependent manner, and that this pathway needs to remain intact for Sema4D-mediated promotion of angiogenesis.

**Figure 3:** RhoA and Akt are necessary for Plexin-B1-mediated activation of NF-κB and promotion of endothelial cell migration and tube formation. A. Immunoblot for phospho-I-κB (top panel) and total I-κB (middle panel) in cells expressing chimeric receptors coding for the extracellular portion of Trk-A fused to the wild-type intracellular segment of Plexin-B1 (wtPB1), Plexin-B1 lacking the PDZ binding motif (ΔPDZ) or Plexin-B1 mutated in the RasGAP domain (RasGAP mut), treated with NGF with and without the Rho inhibitor C3 toxin (C3) and the PI3K inhibitor LY294002 (LY), for the times indicated. GAPDH was used as a loading control (lower panel). B. NF-κB reporter assay performed on control treated HUVEC or HUVEC treated with Sema4D, with or without C3 toxin or LY294002 (LY), with fluorescence expressed as arbitrary units (AU). Error bars represent the standard deviation from three experiments. C. Migration assays on HUVEC towards BSA or Sema4D in the presence of control media, or media containing C3 or LY294002 (LY). Quantification of migration is shown in the bar graph in the lower panel. Error bars represent the standard deviation from six wells (*, p<0.05). D. HUVEC were plated on reconstituted basement membrane material in serum free media and treated with vehicle control (control) or Sema4D, with or without co-treatment with C3 toxin (C3) or LY294002 compound (LY), and examined for formation of capillary tubes. Representative photographs are shown. Quantification of the results observed in the tubulogenesis assay are shown in the right panel (error bars represent the standard deviation from three independent experiments; *, p<0.05).

### Sema4D treatment of HUVEC activates the NF-κB downstream target IL-8, which is necessary for the promotion of angiogenesis

We performed an ELISA on media conditioned by Sema4D treated HUVEC, looking for the presence of IL-8, a known pro-angiogenic downstream target of NF-κB [27]. HUVEC treated with increasing concentrations of soluble Sema4D produced increasing amounts of IL-8, unless when co-treated with the NF-κB inhibitory compound BAY11-7085 (Figure 4A). To determine the biological significance of NF-κB-mediated IL-8 production, we performed a migration assay on HUVEC toward Sema4D, with and without the presence of IL-8 blocking antibody. As expected, Sema4D attracted HUVEC, but this response was attenuated by increasing concentrations of IL-8 blocking antibody (Figure 4B, results quantified in the bar graph, lower panel). Sema4D-induced tube formation in HUVEC growing on reconstituted basement membrane material was also reduced by co-administration of IL-8 blocking antibody (Figure 4C, results quantified in the bar graph, lower panel). These results show that NF-κB-dependent IL-8 production is necessary for Sema4D to promote a pro-angiogenic response in endothelial cells.

**Figure 4:** Sema4D treatment of HUVEC induces NF-κB-dependent production of IL-8, which is necessary to promote angiogenesis. A. ELISA for production of IL-8 in HUVEC treated with the indicated concentrations of Sema4D or 400 ng/ml Sema4D with BAY11-7085 (BAY). Results are expressed as averages in pg/ml. Error bars represent the standard deviation for three independent experiments. B. Cell migration assay for HUVEC migrating towards BSA or Sema4D in the presence of IgG control (IgG) or the indicated concentrations of anti-IL-8 blocking antibody. The results are quantified in the bar graph below as the pixel intensity of the scanned migration assay membrane. Error bars represent the standard deviation from six wells (*, p<0.05). C. HUVEC were plated on reconstituted basement membrane material in control media (BSA) or media containing Sema4D, with IgG control (IgG) or the indicated concentrations of IL-8 blocking antibody and examined for formation of capillary tubes. Representative photographs are shown. Quantification of the results observed in the tubulogenesis assay are shown in the bar graph below (error bars represent the standard deviation from three independent experiments; *, p<0.05).

### NF-κB is activated in endothelium by Sema4D-expressing tumor cells

We have previously shown that many different solid tumors produce Sema4D for the purposes of inducing angiogenesis [16]. Therefore, we wanted to determine if Sema4D production by tumor cells could activate NF-κB in endothelial cells. We infected the HNSCC cell line HN13 with control lentivirus or lentivirus coding for Sema4D shRNA and confirmed protein knockdown in an immunoblot (Figure 5A). We then treated HUVEC with media conditioned by these cell lines and looked for phospho- and total I-κB levels in an immunoblot. A phospho-I-κB response and I-κB degradation was noted in HUVEC treated with media conditioned by control infected HN13 but not in HUVEC treated with media conditioned by Sema4D shRNA infected cells (Figure 5B). To further determine biological significance *in vitro*, we looked for the presence of the p65 NF-κB subunit in the nuclei of endothelial cells lining blood vessels from the tumor stroma of HN13 xenografts implanted into the flanks of nude mice, either control infected or infected with Sema4D shRNA-expressing lentivirus. We observed the presence of p65 in the nuclei of endothelial cells of blood vessels associated with tumors comprised of control infected cells, but less so from the vessels associated with tumors made up of Sema4D shRNA infected cells (Figure 5C). These results are quantified in Figure 5D. Taken together, these results strongly suggest that Sema4D production by tumors activates NF-κB signaling in endothelial cells via Plexin-B1 in order to promote tumor-induced angiogenesis.

**Figure 5:** Sema4D produced by tumor cells activates NF-κB in endothelial cells. A. Immunoblot analysis for Sema4D on lysates from HN13 cells, infected with empty vector control lentivirus (control) or virus coding for Sema4D shRNA (S4DshRNA). GAPDH was used as a loading control (lower panel). B. Immunoblot for phospo- (upper panel) and total (middle panel) I-κB in HUVEC growing in media conditioned by control infected HN13 cells (control, left column) or cells infected with Sema4D shRNA expressing lentivirus (S4DshRNA, right column) for the times indicated. GAPDH was used as a loading control (lower panel). C. Immunofluorescence on tumor xenografts composed of control infected HN13 cells or cells infected with Sema4D shRNA, for CD31 (endothelial cells, red) and p65 (green). The white arrows indicate endothelial cell nuclei. D. The results of the xenograft immunofluorescence expressed as the percentage of p65 positive endothelial cell nuclei counted in 10 high power fields (*, p<0.05).

## Discussion

Most cancers arise from an altered pre-malignant progenitor cell that accumulates genetic damage over time, a factor that contributes to the ability of tumor cells to proliferate inappropriately, avoid natural defenses and acquire resistance to chemotherapy. For this reason, patients often are poor candidates for treatment with traditional cytoreductive therapies but might benefit from the development of anti-angiogenic agents, which instead target the normal, genetically stable endothelial cells that line the vessels that feed the tumor. Indeed, growth and metastasis of solid tumors requires induction of angiogenesis, the creation and remodeling of new blood vessels from a pre-existing vascular network, to ensure the delivery of oxygen, nutrients and growth factors to rapidly dividing transformed cells.

VEGF is an endothelial cell specific growth factor that plays a unique role in the regulation of vascular permeability and physiological and pathological angiogenesis, mainly by acting through its receptor VEGF-receptor 2 (VEGF-R2) on endothelial cells. Many different solid tumors have been shown to produce VEGF, and it has become a tempting target for neutralizing antibodies in the treatment of advanced neoplasms. We have demonstrated that Sema4D is over expressed by many different aggressive carcinomas in a manner analogous to VEGF, and that its activity on Plexin-B1-expressing endothelial cells promotes angiogenesis *in vitro* and *in vivo* [4]. However, the mechanisms of Plexin-B1 signaling continue to be investigated. Our group and others have found that Plexin-B1 activates downstream kinases such as Akt and triggers a G-protein response in Sema4D treated cells [4], [17], [18]. Though the role of NF-κB activation by Akt remains controversial [28], here we show that stimulation of Plexin-B1 signaling induces a Rho and Akt-dependent activation of NF-κB. This effect is independent of the RasGAP activity of Plexin-B1, as a RasGAP mutant receptor construct was still able to induce phosphorylation and degradation of I-κB. It is also a purely Plexin-B1-mediated response and likely does not involve the low-affinity Sema4D receptors CD72 or Plexin-B2 or any components of VEGF signaling, as RNA interference directed at Plexin-B1 blocked Sema4D-mediated NF-κB activation and promotion of a proangiogenic response while having no effect on HUVEC responses to VEGF. Furthermore, stimulation of Plexin-B1 specific signaling through NGF-mediated activation of TrkA/Plexin-B1 chimeric receptors promoted I-κB phosphorylation and degradation.

NF-κB is known to be a crucial mediator of inflammation-induced tumor growth and progression, as well as a strong promoter of oncogenesis and tumor cell survival [29] but its effects in endothelial cells on the promotion of angiogenesis is not well studied. There is conflicting evidence in the literature demonstrating that NF-κB activation can be both pro- and anti-angiogenic, mainly by influencing endothelial cell apoptosis [30], [31]. In our system, we show that NF-κB activation by Sema4D results in promotion of endothelial cell survival, migration and tube formation, but unlike VEGF fails to induce significant cell proliferation. These results led us to speculate that Sema4D might elicit a parallel but slightly more limited angiogenic repertoire in endothelial cells when compared to VEGF. However, we also observed robust Sema4D-dependent stimulation of IL-8. This is a significant finding, as IL-8 is secreted by a variety of cells, including endothelial cells, and plays important roles in inflammation and tumor-induced angiogenesis [21]. Many reports have identified NF-κB as the main transcription factor for stimulating IL-8 promoter activity in response to various stimuli [32]. Our study confirmed that the NF-κB inhibitor BAY 11-7085 abrogated the release of IL-8 induced by Sema4D. Stimulation of the NF-κB/IL-8 axis by Sema4D was crucial, since its blockade attenuated the pro-angiogenic response. We also looked for evidence that tumor cells making Sema4D could induce NF-κB activation in endothelium. We showed *in vitro* that media conditioned by HNSCC cells could induce I-κB phosphorylation and degradation in HUVEC in a Sema4D-dependent manner. *In vivo* we observed p65 translocation in the nucleus of endothelial cells in the tumor stroma when tumors were expressing Sema4D but much less so in vessels associated with tumors where Sema4D had been silenced by shRNA. Taken together these findings suggest that NF-κB induction in endothelial cells is crucial for endothelial cell survival and chemotaxis and that it is induced by tumors producing Sema4D for the purpose of promotion of angiogenesis.

There is at least one report of plexins being involved in activation of NF-κB that also appears to promote cell survival. Catalano *et al.* demonstrated that binding of Semaphorin 6D (Sema6D) to its receptor, Plexin-A1, triggered NF-κB transcriptional activity that supported a pro-survival program in malignant pleural mesothelioma cells [33]. Interestingly, they discovered that unlike for the system studied here, Sema6D-induced NF-κB transcriptional activity was dependent upon Plexin-A1-mediated phosphorylation of VEGF-R2, which associated with Plexin-A1 in a signaling complex [33]. These findings raise the question as to whether or not a co-receptor tyrosine kinase or other signaling protein might be involved in Plexin-B1-mediated activation of NF-κB, particularly since Plexin-B1 itself cannot act as a tyrosine kinase. It has been reported that the tyrosine kinase receptor c-Met cooperates with Plexin-B1 to elicit a Sema4D-mediated signal [2], [3]. Such a possibility is currently being investigated.

In summary, we have provided evidence that Sema4D/Plexin-B1-mediated NF-κB activation and IL-8 production is critical in the generation a pro-angiogenic phenotype in endothelial cells, where it promotes migration and survival. However, further studies likely will be necessary to investigate the mechanisms of signaling. Sema4D production by tumors may represent an alternative angiogenesis pathway and therefore represent another treatment target in addition to anti-VEGF therapy for particularly aggressive cancers.

## Materials and Methods

### Ethics statement

All animal studies were approved by the University of Maryland Office of Animal Welfare, Institutional Animal Care and Use Committee (protocol #: 07-03-01) in accordance with the NIH Guide for the Care and Use of Laboratory Animals.

### Cell culture

Human umbilical vein endothelial cells (HUVEC, ATCC, Manassas, VA) were cultured in Endothelial Cell Medium-2 (EGM-2, Lonza). 293T (ATCC) cells and HN13 cells [34] were cultured in DMEM (Sigma, St. Louis, MO) supplemented with 10% fetal bovine serum (unless otherwise indicated) and 100 units/ml penicillin/streptomycin/amphotericin B (Sigma).

### Purification of soluble Sema4D

Sema4D was produced and purified as described previously [4]. Briefly, the extracellular portion of Sema4D was subjected to PCR and the resulting product cloned into the plasmid pSecTag2B (Invitrogen, Carlsbad, CA). This construct was transfected into 293T cells growing in serum free media. Media containing soluble Sema4D was collected 65 hours post-transfection and purified with TALON metal affinity resin (Clontech Laboratories, Palo Alto, CA) according to manufacturer's instructions. Concentration and purity of the TALON eluates was determined by SDS PAGE analysis followed by silver staining (Amersham Life Science, Piscataway, NJ) and the Bio-Rad protein assay (Bio-Rad, Hercules, CA). In all cases, media collected from cells transfected with the empty pSecTag2B vector were used as control.

### Immunoblot analysis

Cells were lysed in lysis buffer (50 mM Tris-HCl, 150 mM NaCl, 1% NP 40) supplemented with protease inhibitors (0.5 mM phenylmethylsulfonyl fluoride, 1 µl/ml aprotinin and leupeptin, Sigma) and phosphatase inhibitors (2 mM NaF and 0.5 mM sodium orthovanadate, Sigma) for 15 minutes at 4°C. After centrifugation, protein concentrations were measured using the Bio-Rad protein assay (Bio-Rad). 100 µg of protein from each sample was subjected to SDS-polyacrylamide gel electrophoresis and transferred onto a PVDF membrane (Immobilon P, Millipore Corp., Billerica, MA). The membranes were then incubated with the appropriate antibodies. The antibodies used were as follows: Plexin-B1 (Santa Cruz A8); GAPDH (Sigma); phospho-I-κB (Santa Cruz, S.C.-101713); total I-κB (Santa Cruz, S.C.-371); p65 (Neomarkers, Fremont, CA); cleaved caspase 3 (Cell Signaling, Beverly, MA); Sema4D (BD Transduction Labs, BD Biosciences, Palo Alto, CA). Proteins were detected using the ECL chemiluminescence system (Pierce, Rockford, IL). Where indicated, cells were treated with the indicated concentrations of soluble Sema4D, C3 toxin (List Biological Laboratories, Campbell, California), LY294002 (Sigma), LPS (Sigma), or BAY11-7085 (Sigma).

### Nuclear extraction and electrophoretic mobility shift assay (EMSA)

Nuclear extracts were prepared using NE-PER Nuclear and Cytoplasmic extraction kit (Thermo Scientific, Waltham, MA) according to the manufacturer's instructions. EMSAs were performed with the LightShift chemiluminescent EMSA kit (Thermo Scientific). DNA-binding probes for NF-κB (forward: 5′-GATCGAGGGGACTTTCCCTAGC-3′; reverse: 5′-GCTAGGGAAAGTCCCCTCGATC-3′) were annealed and biotin labeled according to the Biotin 3′ End DNA labeling kit (Thermo Scientific). 20 fM labeled oligonucleotides were added to a 20 µl reaction mix consisting of 6 µg of nuclear extracts, DNA binding buffer, Poly (dI-dC), 1% NP-40, and MgCl_2_ in concentrations based on manufacturer's recommendations. For competition assays, unlabeled oligonucleotides were allowed to bind the nuclear extracts (30 min at room temperature) before the addition of labeled probes. Supershift experiments were performed by incubating 1 µg of the anti NF-κB/p65 antibody (Neomarkers) with nuclear extract proteins (6 µg for 30 min at room temperature). The reactions were incubated for additional 20 min with biotin labeled probe. The binding complexes were separated on 6% native DNA polyacrylamide gel, transferred to a positively charged nylon membrane (Thermo Scientific) and then detected using a Chemiluminescent Nucleic acid detection Module (Thermo Scientific) according to the manufacturer's instructions and as previously reported [35].

### Immunofluorescence for p65

HUVEC were grown on sterile glass coverslips in 35-mm six-well plates and treated with 400 ng/ml Sema4D for 60 min. The cells were washed in PBS, fixed in 3% paraformaldehyde for 15 min, and permeabilized in 0.5% Triton X-100 for 5 min. The cells were then incubated with anti-p65 antibody (Neomarkers) diluted 1/200 in PBS with 0.5% BSA at 4°C overnight. After three more washings with PBS, coverslips were placed in a humidity chamber for 1 h and covered with FITC-conjugated anti-rabbit secondary antibody (Sigma, 1∶200 dilution in PBS with 0.5% fetal bovine serum). Coverslips were inverted and mounted onto glass slides with Vectashield containing 4′,6-diamidino-2-phenylindole (DAPI, Vector Laboratories, Burlingame, CA) and viewed using a immunofluorescence microscope.

### NF-κB reporter assay

HUVEC were seeded in 96-well plates at a density of 5×10^3^ cells/well. The following day, the cells were infected with lentiviruses expressing the NF-κB reporter and renilla control (SA Biosciences, Frederick, MD) according to the manufacturer's instructions. After 24 h, the cells were changed to DMEM containing 1% FBS and treated with varying concentrations of Sema4D and the indicated inhibitors (3 µg/ml C3 toxin (List Biological Laboratories) or 50 µM LY294002 (Sigma)) for 18 h, as shown. Firefly and renilla luciferase activities were measured using a Dual-Glo luciferase reporter assay system (Promega, Fitchburg WI), and the ratio of firefly luciferase/renilla luciferase luminescence was calculated as previously described [36]. Assays were performed in triplicate and average and standard deviation calculated.

### Short hairpin (sh) RNA and lentivirus infections

The shRNA sequences for human Sema4D and Plexin-B1 were obtained from Cold Spring Harbor Laboratory's RNAi library (RNAi Codex, http://katahdin.cshl.org:9331/homepage/portal/scripts/main2.pl) [37], [38]. The sequences used as PCR templates for Sema4D shRNA have been previously reported [16]. The sequence used for Plexin-B1 shRNA was 5′- TGC TGT TGA CAG TGA GCG CGC CCA GTA TGT GGC CAA GAA CTA GTG AAG CCA CAG ATG TAG TTC TTG GCC ACA TAC TGG GCA TGC CTA CTG CCT CGG A -3′. Oligos were synthesized (Invitrogen) and cloned into pWPI GW, a Gateway compatible CSCG based lentiviral destination vector. Viral stocks were prepared and infections performed as previously reported [16].

### Migration assays

Media containing 10% FBS (positive control), serum free media containing 0.1% BSA (negative control), or serum free media containing 400 ng/ml of purified Sema4D or 50 ng/ml VEGF, where indicated, were placed in the bottom well of a Boyden chamber to serve as chemoattractants. 50,000 serum starved HUVEC cells infected with control lentivirus, lentivirus coding for Plexin-B1 shRNA, electroporated with empty vector or electroporated with the I-κB super-repressor plasmid [39] were added to the top chamber along with the indicated inhibitors (3 µg/ml C3 toxin, 50 µM LY294002, or 10 µM BAY11-7085) or blocking antibodies (IgG control or 2 µg/ml or 10 µg/ml anti-IL-8 antibody (Lifespan Biosciences)) where indicated. The two chambers were separated by a PVPF membrane (Osmonics, GE Water Technologies, Trevose, PA, 8 µm pore size) coated with 10 µg/ml fibronectin (GIBCO, Carlsbad, CA). The migration assay was then performed as described [20]. Briefly, after 7 h, the chamber was disassembled and the membrane stained with Diff-Quick Stain (Diff-Quick, Dade Behring, Deerfield, Illinois), placed on a glass slide and scanned. Densitometric quantitation was performed with NIH image software and cell migration expressed as pixel intensity. Each experiment was performed six times and average and standard deviation calculated.

### Tubulogenesis assays

HUVEC cells infected with control lentivirus, lentivirus coding for Plexin-B1 shRNA, electroporated with empty vector or electroporated with the I-κB super-repressor plasmid [39], were grown in 35 mm plates coated with 150 µl of Cultrex basement membrane extract (Trevigen, Gaithersburg, MD) and incubated overnight in serum free DMEM or serum free media containing 400 ng/ml of Sema4D or 50 ng/ml VEGF, with or without inhibitors or blocking antibody (10 µM BAY11-7085, 3 µg/ml C3 toxin, 50 µM LY294002, or 2 µg/ml or 10 µg/ml anti-IL-8 antibody, where indicated). Cells were then fixed in 0.5% glutaraldehyde and photographed. Media containing 0.1% BSA served as the negative control. Quantification of results was determined using NIH Image, measuring and summing the length of all tubular structures observed in 10 random fields for three independent experiments.

### [^3^H] Thymidine incorporation assay

[^3^H] thymidine incorporation assay was performed as described elsewhere [40]. Briefly, HUVEC were seeded in 24-well culture plates at 5×10^4^ cells/well and growth-arrested in serum-free medium overnight. Cells were left as controls or incubated with media containing 50 ng/ml VEGF or various concentrations of Sema4D (100–400 ng/ml) for 24 h. 0.5 µCi of [^3^H] thymidine was added to each well, and the cells were incubated for a further 4 h. The final incorporation of [^3^H] thymidine into cells was measured with a liquid scintillation counter (LS-6500; Beckman Instruments, Inc., Fullerton, CA) and results of four independent experiments expressed as average counts-per-minute (cpm) relative to untreated controls.

### Trk/Plexin-B1 fusion proteins

Trk-A/Plexin-B1 fusion proteins were made as previously described [4]. Briefly, the intracellular portion Plexin-B1, with or without the PDZ binding motif, was cut out of the plasmid pCEFL EGFP Plexin-B1 with NheI/NotI and cloned in frame with the N-terminal extracellular and transmembrane portion of the NGF receptor Trk-A in the vector pCEFL-myc. A Trk-A/Plexin-B1 mutant lacking key residues involved in RasGAP activity was generated as previously described [4] using the QuikChange II XL Site-Directed Mutagenesis kit (Stratagene, La Jolla, CA). Mutations were confirmed by sequencing.

### IL-8 ELISA

Confluent HUVECs were serum starved for 4 h, then cultured in serum free medium with or without 100 ng/ml, 200 ng/ml or 400 ng/ml Sema4D or 400 ng/ml Sema4D with 10 µM BAY 11-7085, where indicated, for 12 h. The culture supernatant was collected and used to analyze IL-8 by ELISA (Cytokine Core Facility, University of Maryland School of Medicine). Results are expressed as the average and standard deviation for three independent experiments.

### Tumor xenografts

2×10^6^ HN13 cells infected ex vivo with control lentiviruses and virus coding for Sema4D shRNA were resuspended in 250 µl of serum-free DMEM with an equal volume of Cultrex basement membrane extract (Trevigen) and injected subcutaneously into nude mice. After tumor growth had been recorded, animals were sacrificed and tumors were removed and processed for co-immunofluorescence, as described [41]. Briefly, OCT-embedded 8 µm thick frozen tissue sections were cut onto silanated glass slides, air-dried, and stored at −80°C. They were then thawed, hydrated, fixed and washed in PBS. The following antibodies were used: anti-PECAM (BD Pharmingen; 1∶100 dilution); Anti-p65 (Neomarkers, 1∶100 dilution); Fluorescein anti-rabbit secondary and Texas-red anti-mouse secondary (Vector Laboratories; 1∶200 dilution).

## References

[1] Kolodkin AL, Matthes DJ, Goodman CS (1993). The semaphorin genes encode a family of transmembrane and secreted growth cone guidance molecules.. Cell.

[2] Giordano S, Corso S, Conrotto P, Artigiani S, Gilestro G (2002). The semaphorin 4D receptor controls invasive growth by coupling with Met.. Nat Cell Biol.

[3] Conrotto P, Valdembri D, Corso S, Serini G, Tamagnone L (2005). Sema4D induces angiogenesis through Met recruitment by Plexin B1.. Blood.

[4] Basile JR, Barac A, Zhu T, Guan KL, Gutkind JS (2004). Class IV semaphorins promote angiogenesis by stimulating Rho-initiated pathways through plexin-B.. Cancer Res.

[5] Neufeld G, Shraga-Heled N, Lange T, Guttmann-Raviv N, Herzog Y (2005). Semaphorins in cancer.. Front Biosci.

[6] Ch'ng ES, Kumanogoh A (2010). Roles of Sema4D and Plexin-B1 in tumor progression.. Mol Cancer.

[7] Ohta K, Mizutani A, Kawakami A, Murakami Y, Kasuya Y (1995). Plexin: a novel neuronal cell surface molecule that mediates cell adhesion via a homophilic binding mechanism in the presence of calcium ions.. Neuron.

[8] Tamagnone L, Artigiani S, Chen H, He Z, Ming GI (1999). Plexins are a large family of receptors for transmembrane, secreted, and GPI-anchored semaphorins in vertebrates.. Cell.

[9] Oinuma I, Ishikawa Y, Katoh H, Negishi M (2004). The Semaphorin 4D receptor Plexin-B1 is a GTPase activating protein for R-Ras.. Science.

[10] Tong Y, Chugha P, Hota PK, Alviani RS, Li M (2007). Binding of Rac1, Rnd1, and RhoD to a novel Rho GTPase interaction motif destabilizes dimerization of the plexin-B1 effector domain.. J Biol Chem.

[11] Bishop AL, Hall A (2000). Rho GTPases and their effector proteins.. Biochem J.

[12] Kruger RP, Aurandt J, Guan KL (2005). Semaphorins command cells to move.. Nature Reviews Molecular Cell Biology.

[13] Hayden MS, Ghosh S (2004). Signaling to NF-kappaB.. Genes Dev.

[14] Gupta SC, Sundaram C, Reuter S, Aggarwal BB (2010). Inhibiting NF-kappaB activation by small molecules as a therapeutic strategy.. Biochim Biophys Acta.

[15] Luqman S, Pezzuto JM (2010). NFkappaB: a promising target for natural products in cancer chemoprevention.. Phytother Res.

[16] Basile JR, Castilho RM, Williams VP, Gutkind JS (2006). Semaphorin 4D provides a link between axon guidance processes and tumor-induced angiogenesis.. PNAS.

[17] Perrot V, Vazquez-Prado J, Gutkind JS (2002). Plexin B regulates Rho through the guanine nucleotide exchange factors leukemia-associated Rho GEF (LARG) and PDZ-RhoGEF.. J Biol Chem.

[18] Swiercz JM, Kuner R, Behrens J, Offermanns S (2002). Plexin-B1 directly interacts with PDZ-RhoGEF/LARG to regulate RhoA and growth cone morphology.. Neuron.

[19] Vikis HG, Li W, Guan KL (2002). The plexin-B1/Rac interaction inhibits PAK activation and enhances Sema4D ligand binding.. Genes Dev.

[20] Basile JR, Afkhami T, Gutkind JS (2005). Semaphorin 4D/plexin-B1 induces endothelial cell migration through the activation of PYK2, Src, and the phosphatidylinositol 3-kinase-Akt pathway.. Mol Cell Biol.

[21] Sakamoto K, Maeda S, Hikiba Y, Nakagawa H, Hayakawa Y (2009). Constitutive NF-kappaB activation in colorectal carcinoma plays a key role in angiogenesis, promoting tumor growth.. Clin Cancer Res.

[22] Ozes ON, Mayo LD, Gustin JA, Pfeffer SR, Pfeffer LM (1999). NF-kappaB activation by tumour necrosis factor requires the Akt serine-threonine kinase.. Nature.

[23] Kumanogoh A, Watanabe C, Lee I, Wang X, Shi W (2000). Identification of CD72 as a lymphocyte receptor for the class IV semaphorin CD100: a novel mechanism for regulating B cell signaling.. Immunity.

[24] Masuda K, Furuyama T, Takahara M, Fujioka S, Kurinami H (2004). Sema4D stimulates axonal outgrowth of embryonic DRG sensory neurones.. Genes Cells.

[25] Basile JR, Gavard J, Gutkind JS (2007). Plexin-B1 utilizes RhoA and Rho kinase to promote the integrin-dependent activation of Akt and ERK and endothelial cell motility.. J Biol Chem.

[26] Romashkova JA, Makarov SS (1999). NF-kappaB is a target of AKT in anti-apoptotic PDGF signalling.. Nature.

[27] Rao SK, Pavicevic Z, Du Z, Kim JG, Fan M (2010). Pro-inflammatory genes as biomarkers and therapeutic targets in oral squamous cell carcinoma.. J Biol Chem.

[28] Chen F, Demers LM, Shi X (2002). Upstream signal transduction of NF-kappaB activation.. Curr Drug Targets Inflamm Allergy.

[29] Karin M, Greten FR (2005). NF-kappaB: linking inflammation and immunity to cancer development and progression.. Nat Rev Immunol.

[30] Aurora AB, Biyashev D, Mirochnik Y, Zaichuk TA, Sanchez-Martinez C (2010). NF-kappaB balances vascular regression and angiogenesis via chromatin remodeling and NFAT displacement.. Blood.

[31] Rice J, Courter DL, Giachelli CM, Scatena M (2006). Molecular mediators of alphavbeta3-induced endothelial cell survival.. J Vasc Res.

[32] Abdel-Malak NA, Srikant CB, Kristof AS, Magder SA, Di Battista JA (2008). Angiopoietin-1 promotes endothelial cell proliferation and migration through AP-1-dependent autocrine production of interleukin-8.. Blood.

[33] Catalano A, Lazzarini R, Di Nuzzo S, Orciari S, Procopio A (2009). The plexin-A1 receptor activates vascular endothelial growth factor-receptor 2 and nuclear factor-kappaB to mediate survival and anchorage-independent growth of malignant mesothelioma cells.. Cancer Res.

[34] Ahmed ST, Darnell JE (2009). Serpin B3/B4, activated by STAT3, promote survival of squamous carcinoma cells.. Biochem Biophys Res Commun.

[35] Sultana H, Neelakanta G, Kantor FS, Malawista SE, Fish D (2010). Anaplasma phagocytophilum induces actin phosphorylation to selectively regulate gene transcription in Ixodes scapularis ticks.. J Exp Med.

[36] Sun Q, Zhou H, Binmadi NO, Basile JR (2009). Hypoxia-inducible factor-1-mediated regulation of semaphorin 4D affects tumor growth and vascularity.. J Biol Chem.

[37] Hannon GJ, Conklin DS (2004). RNA interference by short hairpin RNAs expressed in vertebrate cells.. Methods Mol Biol.

[38] Siolas D, Lerner C, Burchard J, Ge W, Linsley PS (2005). Synthetic shRNAs as potent RNAi triggers.. Nat Biotechnol.

[39] Martin D, Galisteo R, Ji Y, Montaner S, Gutkind JS (2008). An NF-kappaB gene expression signature contributes to Kaposi's sarcoma virus vGPCR-induced direct and paracrine neoplasia.. Oncogene.

[40] Yang YH, Wu WK, Tai EK, Wong HP, Lam EK (2006). The cationic host defense peptide rCRAMP promotes gastric ulcer healing in rats.. J Pharmacol Exp Ther.

[41] Amornphimoltham P, Sriuranpong V, Patel V, Benavides F, Conti CJ (2004). Persistent activation of the Akt pathway in head and neck squamous cell carcinoma: a potential target for UCN-01.. Clin Cancer Res.

